# Clinical Efficacy of Persian Medicine Diet Combined with Western Medicine-Based Diet on Proteinuria in Pediatric Nephrotic Syndrome: A Randomized Controlled Clinical Trial

**DOI:** 10.1155/2022/2279209

**Published:** 2022-05-24

**Authors:** Alireza Rahmani, Mohsen Naseri, Masoumeh Mohkam, Monireh Sadat Motaharifard, Mahsa Bakhtiary, Nezhat Shakeri, Reza Ilkhani

**Affiliations:** ^1^Nutrition Research Center, Faculty of Nutrition and Food Sciences, Tabriz University of Medical Sciences, Tabriz, Iran; ^2^Traditional Medicine Clinical Trial Research Center, Shahed University, Tehran, Iran; ^3^Pediatric Nephrology Research Center, Research Institute for Children's Health, Shahid Beheshti University of Medical Sciences, Tehran, Iran; ^4^Mofid Children's Hospital, Shahid Beheshti University of Medical Science, Tehran, Iran; ^5^Department of Biostatistics, School of Par Medicine, Shahid Beheshti University of Medical Sciences, Tehran, Iran; ^6^Department of Traditional Medicine, School of Traditional Medicine, Shahid Beheshti University of Medical Sciences, Tehran, Iran

## Abstract

**Introduction:**

Nephrotic syndrome (NS) is a common chronic kidney disorder during childhood. The most important characteristic of this disease is proteinuria. The Persian medicine (PM) has important dietary recommendations for strengthening the kidney function and treatment of this disease. The aim of this study was to investigate the effect of a diet including PM recommendations and general principles of Western medicine.

**Materials and Methods:**

Twenty children with nephrotic syndrome were randomly divided into intervention and control groups and monitored for one month. The control group received a diet based on the general principles of Western medicine. In the intervention group, in addition to the Western medicine diet, dietary recommendations of PM were also prescribed including the pomegranate (*Cydonia oblonga mill.*), quince (*Cydonia oblonga mill.*), and whole grains (wheat and barley). A 24-hour dietary questionnaire was applied and anthropometric and biochemical indices including spot urine protein (proteinuria), albumin (Alb), urea, creatinine (Cr), total cholesterol (TC), and triglyceride (TG) were measured before and after the study.

**Results:**

The amount of protein intake reduced significantly in the diet of both groups but the differences between the two groups were not significant. Proteinuria reduced significantly in both the Western and PM groups; however, proteinuria was significantly lower in the Persian medicine group compared to the control group. TC and Cr levels reduced significantly in the intervention group, although the changes were not significant compared to the control group.

**Conclusion:**

The results of this study showed that adding dietary recommendations of the Persian medicine to the general rules of the Western medicine diet reduced proteinuria and improved the combat against nephrotic syndrome.

## 1. Introduction

Nephrotic syndrome (NS) is one of the most common chronic renal diseases in children. It is characterized by excessive protein loss in the urine due to glomerular filtration barrier abnormalities [1]. It affects 2–7 per 100,000 children globally and has a male preponderance [2]. It can occur at any age, although it is more frequent in children aged 2–5 years [3]. Kidney Disease Improving Global Outcomes (KDIGO) recommendations describe NS in children as edema, proteinuria (protein >40 mg/m2/h or urine protein-creatinine ratio >2 mg/mg or protein >300 mg/dL or 3+ on urine dipstick), hypoalbuminemia (2.5 g/dl), and hyperlipidemia [4]. Most NS cases are idiopathic, and the most prevalent type of idiopathic NS in children is minimal change disease (MCD), which normally improves after starting corticosteroids but may recur once this medication is discontinued [5].

Proper diet, along with medication, plays an essential role in improving NS and significantly reduces the associated complications and recurrence. Therefore, one of the most critical therapeutic strategies of the Western medicine for treating nephrotic syndrome is the precise adjustment of the patient's diet. Successful treatment of NS with certain diets has been documented in several studies [6–8]. Children with NS have unique nutritional needs based on the etiology and symptoms of the disease [9]. As for the diet of these patients, careful attention should be paid to growth and bone development, preserving renal function, maintaining fluid and electrolyte balance, and managing drug-nutrient interactions [2]. The main focus of the recommended diet for children with nephrotic syndrome is on the accurate calculation of energy and dietary protein and limiting sodium and harmful fats (cholesterol, saturated, and trans-fatty acids) [10]. According to the clinical practice guideline for nutrition in children with chronic kidney disease (KDOQI), the energy of these patients should be calculated accurately because these patients are susceptible to obesity and overweight due to continuous intake of corticosteroids. On the contrary, due to the elevation of urea levels, anorexia, and nausea, they are susceptible to underweight and impaired muscle and bone growth. As a result, their energy consumption should be 100% of EER and carefully calculated and consumed. For this purpose, the equations to estimate energy requirements for children were used [9]. Moreover, the protein requirement of the pediatric group should be 100–140% of the dietary reference intake (DRI) for chronic kidney disease stage 1–3 (CKD1-3). At this dose, despite compensating for the amount excreted through urine, excess protein intake does not put extra strain on the kidneys [10]. Edema is an important manifestation in children with nephrotic syndrome, and the main approach to control it is sodium restriction in the range of 1500 to 2400 mg per day depending on age [10]. Due to lipid profile disorders in many patients with nephrotic syndrome, all individuals are advised to limit their dietary sources of saturated and trans-fatty acids [9].

Although the effectiveness of medicines and diets based on the Western medicine has already been proven, there are still some limitations. Delayed recovery and response to Western medicine drugs and diets have led to more consumption of corticosteroids, which have many side effects such as obesity and diabetes. Recurrence of the disease after drug discontinuation is relatively common in these children.

Nowadays, there is a widespread tendency to use complementary and alternative medicine (CAM) therapies. It has been shown that the use of integrated methods of CAM and Western medicine can lead to better treatment results [11–18]. Persian medicine (PM), as one of the CAM methods, provides different strategies for the prevention and treatment of diseases. Dietary recommendations are an essential part of these strategies. As mentioned in Persian medical sources, the first step of treatment is nutritional modifications [19].

The clinical symptoms of NS are very similar to the symptoms of kidney weakness in the Persian medicine. According to the main sources of PM, kidney weakness is a disorder in which the kidneys cannot hold large molecules (such as some proteins), so it is excreted in the urine. The quince (*Cydonia oblonga mill.*), pomegranate (*Punica granatum*), and whole grains (especially wheat and barley), in different forms, are the recommended foods for nephrotic syndrome patients in PM. It is believed that these food items have some medicinal properties and nutritional values, which can promote the kidney's health [19–21].

In Western medicine, the effects of some foods and supplements on nephrotic children have been studied [3, 7, 22]. However, if the dietary recommendations of PM are helpful in controlling and treating the disease, these interventions can be added to the treatment protocol of children with nephrotic syndrome to achieve better clinical results.

Therefore, this study was conducted to evaluate the efficacy and safety of the integrated Persian medicine-based diet and Western medicine in improving urinary protein loss in children with nephrotic syndrome.

## 2. Materials and Methods

### 2.1. Study Setting and Design

A randomized parallel-group clinical trial was conducted in Mofid Hospital affiliated with Shahid Beheshti University of Medical Sciences, Tehran, Iran. The duration of the study was one month.

### 2.2. Participants

The participants were 20 outpatient children (14 boys and 6 girls) aged 2–12 years recruited from the Pediatric Nephrology Clinic of Mofid Hospital. A pediatric nephrologist confirmed the diagnosis of minimal change nephrotic syndrome before the participants were recruited.

Children with a body mass index (BMI) of 5–85th percentile and CKD 1–2 that were willing to join the study were included. The children were excluded from the study if they had any severe congenital or inherited diseases, heart failure, advanced renal failure, hypo or hyperthyroidism, and severe inflammatory diseases such as lupus erythematosus, diabetes mellitus, and severe edema. All patients had a history of proteinuria recurrence.

### 2.3. Interventions

The Western medicine regimen was calculated individually for patients in both groups and explained to them.

In the intervention group, a Western medicine-based diet was given in accordance with the principles of Persian medicine. Three simple foods were added to the diet of this group, which included one tablespoon (Tbsp) of quince sauce after each meal three times a day (TDS), one Tbsp of pomegranate paste before each meal TDS, and one Tbsp of whole-wheat powder (*Savigh*) as a snack once a day (with a cup of water or milk). To adjust the diets of both groups, attention was paid to consider similar mean energy and macronutrients for the two groups with no significant difference. The individuals in both groups were carefully followed, and laboratory tests were measured before and four weeks after the intervention in all participants. Both groups received routine drug treatments for NS during the study period (Prednisolone, Enalapril).

### 2.4. Primary and Secondary Outcomes

The primary outcome measures of this study were spot urine protein (UPr) and urine protein/creatinine ratio (UPCR). Secondary outcome measures were urine creatinine (UCr), serum albumin, urea, total cholesterol (TC), and triglyceride (TG).

### 2.5. Biochemical Assessment

Following 10–12 hr of fasting, 10 ml venous blood was collected from the participants in the beginning and at the end of the study. The serum was separated from whole blood by centrifugation at 3000 rpm for 7 minutes (Orum Tadjhiz centrifuge, Iran) at room temperature. The sera were stored at −70°C until assay. The patients were asked not to engage in physical activity for 30 minutes before blood sampling.

Spot urine protein and creatinine were determined by colorimetric methods using an Olympus 5400 series analyzer (Olympus Diagnostics, Dallas, TX). Although 24-hour urine collection is the gold standard for estimating proteinuria, children sometimes do not accept to do it because it is cumbersome. According to previous studies, spot urine protein-creatinine ratio (UPCR) is a reliable index to measure urine protein, which is more acceptable and takes less time [23, 24]. Serum TG and TC levels were tested using commercially available diagnostic kits (all purchased from Pars Azmoon Co. Ltd., Iran). Biochemical solutions were used to measure albumin creatinine, urea, and uric acid levels.

### 2.6. Dietary Evaluation and Anthropometric Indices

The participants underwent a standard clinical assessment comprising a medical history and physical examination. To assess the nutritional intake of the patients, they were asked to complete a 24-hour recall questionnaire for three days (two weekdays and one weekend). The results were analyzed using the Nutritionist IV (First Databank Inc., Hearst Corp., San Bruno, CA) modified for Iranian foods to calculate total energy, carbohydrate, protein, and fat. A stadiometer with 0.1 cm accuracy was used to measure the height while standing near a wall. The weight was measured using a weighing scale (Seca, Hamburg, Germany) to the nearest 0.1 kg with minimal clothing without shoes.

### 2.7. Follow-up

All patients were requested not to change their physical activity and diet during the study period. To ensure compliance with the intervention protocol, they were asked to return to the clinic after two weeks to receive the remaining supplements and monitoring for any probable adverse events. The researcher's phone number was provided to the patients for a better follow-up.

### 2.8. Sample Size Calculation

The sample size study was calculated based on the primary data of urinary protein excretion obtained from a previous study (D.H.Sandberg, LANCET, 1977). Considering a confidence interval of 95% and a power of 80% and using the standard formula for clinical trials ((*σ*_1_^2^+*σ*_2_^2^)(*Z*_*α*/2_+*Z*_*β*_)^2^/(*μ*_1_ − *μ*_2_)^2^), the sample size was calculated at eight patients. Considering a 20% drop, 10 subjects were considered for each group (20 patients in total).

### 2.9. Randomization

The patients included in the study were randomized into two groups by a simple randomized method using the RAS (random allocation software) and were followed for one month. Since corticosteroids can be a confounder for the results of dietary intervention, patients were matched in the two groups in terms of the prednisolone dose (0/5–0/99, 1–1/49, and 1/5–2 mg/kg/d).

### 2.10. Statistical Analysis

The data were analyzed using the IBM SPSS software version 23 (IBM SPSS Statistics, Armonk, USA). To describe quantitative data, variables with a normal distribution are presented as mean ± SD and mean difference (95% CI) and variables with a non-normal distribution are reported as median (IQB) and median difference. The normal distribution of the data was evaluated using the Shapiro–Wilk test. Independent samples *t*-test and Mann–Whitney *U* test were applied to variables with anormal and non-normal distribution values to examine the differences between intervention and control groups at baseline, respectively. To assess between-group differences of qualitative variables, Fisher's exact test, and chi square test were applied, as appropriate. Paired samples *t*-test and Wilcoxon signed-rank test were used to investigate within-group changes in variables with a normal and abnormal distribution, respectively. Analysis of covariance (ANCOVA) was used to eliminate the impact of confounding factors (i.e., baseline values, protein intake, and BMI) on the result. For this reason, two distinct models were sued, including baseline values (model 1) and baseline values, protein intake, and BMI (model 2). The level of significance was set at 0.05. Missing data were removed from the final analysis.

### 2.11. Ethical Considerations

The study protocol was explained to the participants and informed consent was obtained from them.

The study protocol was approved by the Research Ethics Committees of Shahed University in accordance with the Declaration of Helsinki (IR.SHAHED.REC.1400.064).

The study was also registered in the Iranian Registry of Clinical Trials (IRCT20200411047027N20. The personal information of enrolled participants was collected and maintained confidentiality by encoding systems. At the end of the study, the results of biochemical tests were given to the participants.

## 3. Results

The process of recruitment and randomization is illustrated in Figure 1. A total of 65 patients presenting to the Pediatric Nephrology Clinic of Mofid Hospital were assessed for eligibility. According to the inclusion and exclusion criteria, 20 patients were randomly allocated to intervention and control groups. One patient withdrew from the intervention group due to parents' hesitation to continue the study and was excluded from the final analysis.

The demographic characteristics of both groups are shown in Table 1. At the beginning of the study, there was no significant difference in age, sex, weight, height, and the dose of prednisolone between the two groups. However, the intervention group had a significantly higher mean BMI compared to the control group.

As shown in Table 2, there was no significant difference in the amount of energy and macronutrients (carbohydrate, protein, and fat) between the two groups at the beginning and in the end of the study. However, due to the diet adjustment according to the KDOQI guideline, the amount of protein consumed by both groups was significantly lower at the end of the study compared to the initial amount (*p*=0.032, *p*=0.038).

Changes in biochemical parameters are presented in Table 3. Before the intervention, there were no significant differences in UPr (*p*=0.990), UPCR (*p*=0.802), UCr (*p*=0.919), Alb (*p*=0.685), urea (*p*=0.828), TC (*p*=0.072), and TG (*p*=0.744) between the two groups. At the end of the study, within-group analysis showed a significant decline in UPr and UPCR in the intervention (*p*=0.028) and control (*p*=0.028) groups. In addition, TC (*p*=0.050) decreased significantly in the intervention group. According to paired sample *t*-test, other indicators did not show substantial changes within each group. After adjusting for baseline values, changes in protein intake, and BMI, a between-group analysis was performed (ANCOVA test), and changes in UPr (*p*=0.014) and UPCR (*p*=0.007) were statistically significant compared to the placebo group. No significant side effects were reported during the study period.

A significant difference was found in the percentage of changes in UPr and UPCR between the two groups (Figure 2).

## 4. Discussion

To the best of our knowledge, the present study is the first study that evaluated the efficacy of PM recommendations in nephrotic syndrome. According to the findings, protein excretion and urine protein/creatinine ratio reduced significantly in both the Western and PM groups. However, both indices were significantly lower in the PM group. Considering that the drugs used by patients (prednisolone) were matched between the two groups at the beginning of the study and other confounding factors (protein intake, BMI, and initial values) were adjusted in the final analysis, this significant difference can be attributed to the difference in the diet. As stated in the introduction, the clinical symptoms of NS are very similar to the symptoms of kidney weakness in PM in that the kidneys are unable to work effectively, resulting in protein loss in the urine. In PM, several dietary recommendations have been proposed to cure this condition, including pomegranate paste, quince sauce, and whole wheat.

Pomegranate paste is the first food suggested in PM to combat nephrotic syndrome. The primary sources of the Iranian traditional medicine reported that pomegranate paste reduced protein excretion by strengthening the kidney tissue [19–21]. In previous studies, pomegranate juice has shown nephroprotective effects through stabilizing and improving the kidney function of rats [25]. In addition, the use of pomegranate extract effectively maintains normal total protein levels in rats with acute renal failure [26]. Pomegranate has powerful antioxidant and anti-inflammatory capabilities to the extent that it is referred to as a “superfruit” by some [27]. The antioxidant and anti-inflammatory properties of this fruit are the reasons for its nephroprotective effects on the kidneys. These properties are most likely due to the presence of several bioactive components, including oleanolic acid (OA), ursolic acid (UA), gallic acid (GA), and punicalagin [28]. In a study in 2020, Y. Seo et al. found that punicalagin (a key polyphenol found abundantly in the pomegranate) suppresses extracellular signal-regulated kinase (ERK), mitogen-activated protein kinase (MAPK), and nuclear factor kappa B (NF-*κ*B) pathways, thus decreasing inflammation in the kidneys [29].

Quince is another PM recommendation for strengthening the kidneys. The quince, like the pomegranate paste, is rich in flavonoids and antioxidants, which helps to improve glomerular dysfunction and decrease urine protein excretion [30]. Previous studies have recommended the use medicines that block the renin-angiotensin axis in children with steroid-resistant nephrotic syndrome (SRNS) [31–33]. In children with SRNS, angiotensin-converting enzyme inhibitors (ACEIs) have been shown to reduce proteinuria with a response rate of 40–50% [34, 35]. Through a similar mechanism, the quince reduces the concentrations of renin and angiotensin and increases the nitric oxide level, thereby lowering systolic blood pressure [33]. According to the W.t. Zhou et al., this impact is dosage-dependent, and its effect is similar to captopril at the maximum recommended dose [33].

Another important recommendation of the traditional medicine diet is whole wheat, one of the richest sources of bran and dietary fiber. In a meta-analysis study, D Aune et al. found that whole grains consumption reduced the risk of cardiovascular disease, cancer, and all-cause and cause-specific mortality [36]. In addition, whole grains can positively affect the kidney function and improve CKD, whereas refined grains are adversely associated with eGFR [37]. One of the mechanisms for this phenomenon could be the beneficial effects of whole wheat on the microbiome. The gut microbiota may have a protective or detrimental effect on the kidney either directly or indirectly by influencing the primary risk factors for the development and progression of CKD, including inflammation, diabetes, hypertension, and proteinuria [38]. Patients with nephrotic syndrome have significantly different alpha and beta diversity, as well as lower gut microbiota-derived short-chain fatty acids (SCFA) [39]. On the contrary, early treatment of children with nephrotic syndrome boosts the number of SCFA-producing gut bacteria [40]. Daily use of whole wheat promotes the growth of intestinal microbiota, increases SCAF production, and improves gastrointestinal health [41, 42].

The findings of the present study suggest that pomegranate, quince, and barley compounds can be added to the diet of children with nephrotic syndrome.

Previous research has linked protein excretion to hyperlipidemia [43, 44]. Proteinuria reduces serum albumin levels, which causes the liver to produce more albumin to maintain the plasma colloid osmotic pressure. Because albumin is synthesized along with lipoproteins, serum cholesterol, and triglycerides rise [45, 46]. Reduced lipoprotein lipase (LPL) synthesis [47], VLDL deficiency [48, 49], decreased LDL receptor (LDLR) sensitivity, and impaired clearance of apoB-100 [50–52] are additional mechanisms contributing to the increase in TG, apoB-containing lipoproteins (such as VLDL, IDL, and LDL), Lp (a), and total cholesterol in nephrotic syndrome [46]. As a result, throughout the treatment process, by lowering proteinuria, serum albumin levels increase in the first phase, and the amount of lipoproteins decreases in the next step. According to the findings of this study, spot urine protein dropped significantly in the group receiving the traditional diet. Although serum albumin increased and cholesterol decreased, these changes were not statistically significant in between-group or within-group comparison. The short period of the research may be the reason for the lack of significance of these changes.

### 4.1. Strengths and Limitations of the Study

This clinical trial had several strengths. Since the intervention group's diet contained a combination of the most important dietary recommendations of traditional medicine and the general principles of Western medicine diet and the control group only received a diet based on modern medicine, it was possible to compare the two groups. In addition, a renal diet was planned for all patients based on the individual characteristics of the participants; thus, protein excretion decreased significantly in both groups. Random allocation and matching the two groups in terms of their drugs (prednisolone) were other advantages.

Nevertheless, the present study was limited in some ways. Since no similar study was conducted in children with nephrotic syndrome, the shortest duration of the study was considered.

The best way to calculate energy requirements is using indirect calorimetry. Due to difficult access and insufficient facilities, we used the proposed standard formulas to estimate participants' energy. Since our intervention was in the form of a dietary change and it was not possible to design a placebo for the control group, patients were not blind to the intervention. However, to solve this problem, the control and intervention groups were sampled in two separate places so that patients were not aware of the difference in diet given to the other group. Because of funding limitations, we could not evaluate anti-inflammatory and antioxidant factors. Although the sample size was calculated according to the most similar study available, it is necessary to conduct subsequent studies in larger sample sizes, and also in adult patients, to confirm the results. These limitations should be considered in the interpretation of the findings and also in future studies.

## 5. Conclusion

Nephrotic syndrome is a complex pediatric kidney disease requiring attention to nutrition and pharmacologic therapies. Recently, many attempts have been made to use alternative medicine to treat various kidney diseases. Diet management may be extremely helpful in the treatment of these diseases. This study suggests that a combination of the Persian medicine-based diet and Western medicine principles optimizes proteinuria and improves NS. However, the present study was conducted on a relatively small sample size. Further studies in larger sample sizes with longer treatment and follow-up times are required to confirm the results.

## Figures and Tables

**Figure 1:** Flow diagram of the recruitment and randomization process.

**Figure 2:** Effect of combined diet on UPr and UPCR in two study groups: (a) Percentage of UPr changes. (b) Percentage of UPCR changes. Values are mean of percentage of change ± SEM. UPr = spot urine protein; UPCR = urine protein/creatinine ratio. ^*∗*^ANCOVA test (adjusted for BMI, and changes in protein intake).

**Table 1:** Baseline characteristics of participants.

Variables	Intervention group (*N* = 9)	Control group (*N* = 10)	*P* ^a^
Age (year)	10.89 ± 1.47	8.10 ± 1.20	0.158^a^
Weight (kg)	38.89 ± 4.41	30.70 ± 5.16	0.250^a^
Height (cm)	1.34 ± .09	1.28 ± .07	0.617^a^
BMI (kg/m^2^)	20.60 (4.17)	17.36 ± .97	0.043^a^
Sex			0.350^b^
Boy	5 (55.6)	8 (80.0)	
Girl	4 (44.4)	2 (20.0)	
Intake of drugs			
Prednisolone (0/5-0/99 mg/kg/d)	3 (33.3)	3 (30.0)	1.000^b^
Prednisolone (1-1/49 mg/kg/d)	3 (33.3)	5 (50.0)	0.650^b^
Prednisolone (1/5-2 mg/kg/d)	3 (33.3)	2 (20.0)	0.628^b^
Enalapril (5 mg/d)	4 (44.4)	5 (50.0)	1.000^b^

Mean ± SD and median (IQR) are presented for normally and not normally distributed measures, respectively. Frequency (percentage within subgroup) has been used for qualitative variables. BMI = body mass index; SD = standard deviation; IQR = interquartile Range. *P*^*a*^ = independent samples *t*-test. *P*^*b*^ = Fisher exact test.

**Table 2:** Dietary intake of participants.

	Intervention group (*N* = 9)	Control group (*N* = 10)	MD	*P*
Energy (Kcal)				
Baseline	1554.44 ± 123.36	1402.00 ± 175.21	152.44 (−309.41, 614.30)	0.496^b^
End	1497.78 ± 114.71	1456.00 ± 124.12	41.77 (−317.42, 400.98)	0.386^c^
MD (95% CI)	56.66 (−12.72, 126.06)	−54.00 (−249.12, 141.12)		
*P*^*a*^	0.096	0.547		
Carbohydrate (gr)				
Baseline	213.33 ± 16.91	198.90 ± 14.49	14.43 (−32.29, 61.16)	0.523^b^
End	205.67 ± 15.74	192.70 ± 16.47	12.96 (−35.37, 61.30)	0.745^c^
MD (95% CI)	7.66 (−33.36, 48.70)	6.20 (−33.82, 46.22)		
*P*^*a*^	0.678	0.734		
Protein (gr)				
Baseline	46.44 ± 4.54	51.10 ± 3.83	−4.65 (−15.98, 6.67)	0.398^b^
End	37.11 ± 2.89	40.60 ± 3.28	−3.48 (−12.82, 5.84)	0.622^c^
MD (95% CI)	9.33 (1.03, 17.63)	10.50 (0.71, 20.28)		
*P*^*a*^	0.032	0.038		
Fat (gr)				
Baseline	56.67 ± 4.54	53.60 ± 4.08	3.06 (−9.77, 15.91)	0.683^d^
End	61.33 ± 3.59	57.90 ± 4.94	3.43 (−9.68, 16.55)	0.660^c^
MD (95% CI)	−4.66 (−18.21, 8.87)	−4.30 (−16.11, 7.51)		
*P*^*a*^	0.450	0.033 (P^e^)		

Values are presented as Mean ± SD, and mean difference (95% CI) are presented for all the variables. MD = mean difference; SD = standard deviation; CI = confidence interval; ANCOVA = analysis of covariance. *P*^*a*^ = paired samples *t*-test. *P*^*b*^ = independent samples *t*-test. P^*c*^ = *ANCOVA test, adjusted for baseline values. P*^*d*^ = *Mann–Whitney U test. P*^*e*^ = *Wilcoxon* signed-ranked test.

**Table 3:** Proteinuria and biochemical parameters of the study participants throughout study.

	Intervention group (*N* = 9)	Control group (*N* = 10)	MD	*P*
UPr (mg/dl)				
Baseline	157.00 ± 33.98	156.46 ± 27.67	.54 (−91.15, 92.23)	0.990^b^
End	98.31 ± 22.50	140.32 ± 23.03	−42.00 (−110.23, −26.21)	0.018^c^, 0.014^d^
MD (95% CI)	58.68 (8.33, 109.04)	16.14 (2.21, 30.06)		
*P*^*a*^	0.028	0.028		
UCr (mg/dl)				
Baseline	55.41 ± 9.11	54.28 ± 6.56	1.13 (−22.20, 24.47)	0.919^b^
End	46.46 ± 8.93	54.22 ± 6.30	−7.75 (−30.46, 14.95)	0.245^c^, 0.072^d^
MD (95% CI)	8.94 (−9.03, 26.93)	0.05 (−2.43, 2.54)		
*P*^*a*^	0.284	0.959		
UPCR				
Baseline	2.64 ± 0.25	2.72 ± 0.16	−.07 (−.70, 0.55)	0.802^b^
End	1.94 ± 0.21	2.47 ± 0.12	−.525 (−1.03, −0.01)	0.015^c^, 0.007^d^
MD (95% CI)	0.70 (0.20, 1.19)	0.25 (0.10, 0.39)		
*P*^*a*^	0.011	0.004		
Alb (mg/dl)				
Baseline	3.77 ± 0.37	3.90 ± 0.19	−0.12 (−0.74, 0.50)	0.685^b^
End	4.01 ± 0.08	3.80 ± 0.24	0.21 (−0.36, .78)	0.383^c^, 0.765^d^
MD (95% CI)	−0.23 (−0.74, 0.27)	0.10 (−0.47, 0.67)		
*P*^*a*^	0.321	0.703		
Urea (mg/dl)				
Baseline	31.44 ± .22	30.60 ± 2.80	0.84 (−7.22, 8.91)	0.828^b^
End	29.00 ± 2.07	27.30 ± 2.29	1.70 (3.11, −4.87)	0.600^c^, 0.957^d^
MD (95% CI)	2.44 (−1.66, 6.55)	3.30 (−1.28, 7.88)		
*P*^*a*^	0.207	0.138		
TC (mg/dl)				
Baseline	227.89 ± 26.65	165.50 ± 19.39	62.38 (−6.15, 130.93)	0.072^b^
End	194.78 ± 16.01	163.90 ± 22.67	30.87 (−28.93, 90.69)	0.267^c^, 0.148^d^
MD (95% CI)	33.11 (−0.04, 0.66.18)	1.60 (−12.81, 16.01)		
*P*^*a*^	0.050	0.807		
TG (mg/dl)				
Baseline	149.00 ± 19.77	159.80 ± 25.14	−10.80 (−79.36, 57.76)	0.744^b^
End	134.33 ± 14.22	158.80 ± 27.44	−24.46 (−91.94, 43.00)	0.501^c^, 0.114^d^
MD (95% CI)	14.66 (−33.90, 63.23)	1.00 (−41.34, 43.34)		
*P*^*a*^	0.506	0.959		

Mean ± SD, and mean difference (95% CI) are presented for normally distrusted data; median (IQB) and median differences are presented for data not normally distributed. UPr = spot urine protein; UCr = urine creatinine; UPCR = urine protein/creatinine ratio; Alb = albumin; TC = total cholesterol; TG = triglyceride; MD = mean difference; SD = standard deviation; IQR = interquartile Range; ANCOVA = analysis of covariance. *P*^*a*^ = paired samples *t*-test. *P*^*b*^ = independent samples *t*-test. *P*^*c*^ = *ANCOVA test, adjusted for baseline values. (Model 1). P*^*d*^ = *ANCOVA* test, adjusted for baseline values, changes in protein intake, and BMI. (Model 2).

## Data Availability

The datasets generated during this study will be available via the corresponding author on a reasonable request.
